# Effects of Patellofemoral Pain Syndrome on Changes in Dynamic Postural Stability during Landing in Adult Women

**DOI:** 10.1155/2022/7452229

**Published:** 2022-05-10

**Authors:** Chanki Kim, Seunghyeok Yeom, Seji Ahn, Nyeonju Kang, Kiwon Park, Kyoungkyu Jeon

**Affiliations:** ^1^Department of Human Movement Science, Incheon National University, Incheon, Republic of Korea; ^2^Functional Rehabilitation Biomechanics Laboratory, Incheon National University, Incheon, Republic of Korea; ^3^Division of Sport Science, Incheon National University, Incheon, Republic of Korea; ^4^Sport Science Institute, Incheon National University, Incheon, Republic of Korea; ^5^Health Promotion Center, Incheon National University, Incheon, Republic of Korea; ^6^The Department of Mechatronics Engineering, Incheon National University, Incheon, Republic of Korea

## Abstract

**Background:**

This study investigated the effects of lower limb movements on dynamic postural stability (DPS) during drop landing in adult women with patellofemoral pain syndrome (PFPS).

**Methods:**

Thirty-eight adult women were recruited and divided into two groups, the PFPS group and the control group. The study participants performed a single-leg drop landing from a 30 cm box, and their lower limb movements and DPS were measured. Differences between groups were examined using independent sample *t*-tests. In addition, stepwise multiple linear regression was used to examine the kinematic parameters that contribute to the DPS.

**Results:**

The PFPS group had significantly lower hip flexion, internal rotation, knee flexion, ankle external rotation, pelvic oblique, tilt, rotation, and higher hip abduction, knee valgus, and ankle plantarflexion. In terms of DPS, the PFPS group had a significantly higher anteroposterior and a lower mediolateral than that of the control group. In the control group, regression analysis revealed a controlled anteroposterior using knee flexion, while the PFPS group controlled mediolateral through ankle plantarflexion.

**Conclusions:**

Patients with PFPS experienced more shock on their knee joint during landing than patients in the control group with greater anteroposterior instability and lower mediolateral instability.

## 1. Introduction

The patellofemoral pain syndrome (PFPS) is a disease that is characterized by continuous pain around the anterior knee. It is caused by several factors, such as excessive use of the knee joint, cartilage injury, increased *Q*-angle, vastus medialis weakness, and patellar misalignment and instability [1–3]. PFPS are reported to affect one out of every six physically active individuals, and affected individuals tend to engage in less physical activity due to the pain [4]. A study that followed up patients diagnosed with PFPS as teenagers for 10 years discovered that 91% of the patients suffered functional impairment, local tenderness, patellar femoral friction, and faced difficulty bending the knees due to continuous knee pain [5].

Because women have a wider pelvis in relation to their femoral length, they are twice as likely as men to develop PFPS [6]. Consequently, knee and hip flexion causes excessive adduction and internal rotation, reducing the patellofemoral joint contact area [7]. Furthermore, women have a weaker quadriceps femoris, with a larger *Q*-angle than men, which delays the activation of the vastus medialis in a dynamic situation while increasing the lateral glide of the patella and knee joint pressure, resulting in pain [3, 8].

Women are reported to experience more patellofemoral stress while running, jumping, landing, and climbing stairs due to the increased load during knee flexion as a result of these structural features [1, 9]. Landing, a common task performed in daily life and sports, generates shock that is 2–3 times greater than body weight [10], and the knee joints play an important role in shock absorption during landing, absorbing approximately 41% of the total shock [11]. However, small hip flexion and large internal rotation during landing direct substantial shock onto the knee joints, and the consequently greater patellofemoral stress increases the risk of an injury [12] Women with PFPS put more strain on the patellofemoral joint during single-leg squats and landing, due to excessive knee abduction, increasing their risk of anterior cruciate ligament (ACL) injury and arthritis [13–16].

As described here, the assessment of lower limb movement and balance during a dynamic task, such as a single-leg squat or landing, is a valid method for predicting the risk of potential knee injuries [17, 18]. Patients with PFPS have been reported to have unstable landing patterns during double-leg landing, compared to their healthy counterparts [19]. These patients try to reduce knee pain by increasing hip flexion. However, they have a greater tibial internal rotation moment and an anteriorly displaced center of pressure (COP) [19]. Among the various methods for assessing dynamic postural stability [20, 21], dynamic posture stability (DPS) can be used as an indicator of the ability to maintain balance during the transition from a dynamic to a static state upon landing [22].

Landing motion is a common activity in daily life, and previous research has primarily focused on the knee joint during landing. Because women with PFPS may experience changes in the movement patterns of their entire lower limbs during landing due to structural differences, not only the knee joint but also the ankle joint and hip joint must be examined [13, 23, 24]. Furthermore, studies comparing the factors of dynamic stability during landing between patients with PFPS and healthy individuals, as well as identifying the specific dynamic factors that affect the DPS, are lacking. This study is aimed at comparing the kinematic features of major lower limb joints during single-leg landing between adult women with PFPS and their healthy counterparts, as well as to identify the specific kinematic parameters that contribute to the DPS via regression analysis, to present foundational data for developing desirable landing strategies for patients with PFPS. The hypotheses of this study are as follows. First, during single-leg drop landing, the PFPS group will have a significant difference in the angles of the hip and knee joints in the frontal plane compared to the control group. Second, the kinematic parameters affecting DPS will also appear differently.

## 2. Materials and Methods

### 2.1. Study Participants

Thirty-eight women aged 20–29, with no history of lower limb joint injuries in the previous 6 months, other than PFPS, were enrolled. The participants were divided into two groups based on their orthopedic diagnosis of PFPS: the PFPS group (*n* = 19) and the control group (*n* = 19). This study was approved by the Institutional Review Board of the Incheon National University (INUIRB No. 7007971-201801-001). This experiment was conducted according to the Declaration of Helsinki (1964). The participants provided informed consent after receiving sufficient explanations regarding the study contents and procedures.  Table 1 presents the physical characteristics of the participants.

### 2.2. Procedures

Drop landing is based on a study by Orishimo et al. [25], participants were instructed to perform a drop landing from a 30 cm box by slowly shifting their body weight anteriorly and landing in a free fall. Landing outside the ground force plate or stumbling on landing were considered failed attempts, and measurements were repeated in such cases. Because the left side was affected in the PFPS group, both groups were instructed to land on their left leg. To prevent injury, the participants performed 10 minutes of warm-up and practiced drop landing for 15 minutes before beginning the measurement. To ensure accurate measurements, all participants performed a single-leg drop landing and maintained balance for at least 5 seconds after landing. To improve accuracy, the analysis used the average values of three repeated measurements of successful attempts.

### 2.3. Data Analysis

#### 2.3.1. Motion Analysis

During a drop landing, eight video analysis cameras (6 Eagle & 2 Raptor Camera System, Motion Analysis Corp., Santa Rosa, CA, USA) and one ground force plate (OR6-5-2000, AMTI Inc., Watertown, MA, USA) were used to collect kinematic and kinetic data from lower limb joints. The video analysis cameras were installed around the participant (anteroposterior and mediolateral), such that the entire range of motion with reference to the reference coordinates could be captured. Segment axis systems were established with the *x*-axis designated as the mediolateral direction of drop landing, the *y*-axis as the anteroposterior direction, and the *z*-axis as the vertical direction off the ground. The equipment was calibrated to establish spatial coordinates. To measure the anatomical static posture, 19 reflective markers were attached around the major lower limb joints using Helen Hayes Marker Set [26]. The remaining 15 markers were used to take measurements during the drop landing task after four markers attached to the knee joints and the medial aspect of the ankle joints were removed (Figure 1).

Using Cortex 5 (Motion Analysis Corp., Santa Rosa, CA, USA), we processed all kinematics and kinetic data. The data was sampled at 120 frames per second. For data processing, it was smoothed using digital filtering (Butterworth Low-Pass Digital Filtering) method to remove noise errors, the point of peak vertical GRF was analyzed, and a rigid body system was used for the analysis (Figure 2). The cut-off frequency was set at 10 Hz to minimize error during data processing. We synchronized the data using an analog-digital converter (A/D convertor, NI-USB 6218, National Instruments, Hungary) for measurement and analysis to align the time points for all data.

#### 2.3.2. Dynamic Postural Stability Index (DPSI)

GRF values were established with the xGRF designated as the mediolateral direction of drop landing, the yGRF as the anteroposterior direction, and the zGRF as the vertical direction off the ground. DPSI was computed based on the study by Wikstrom et al. [22]. The stability was calculated with reference to three directions (anteroposterior, mediolateral, and vertical). The stability is a mean square deviation that assesses variation around zero rather than a standard deviation that assesses variation around the mean. The medial-lateral stability index (MLSI) and anterior-posterior stability index (APSI) assess variation around zero along the mediolateral and anteroposterior axes of the force plate, and the vertical stability index (VSI) assesses the variation in vertical GRF along the vertical axis of the force plate standardized with the participant's body weight. To ensure the accuracy of the DPSI analysis, data was collected for 3 seconds from the point of initial contact with the ground for the calculation [22, 27].

(1) $$\begin{array}{c} \text{MLSI}=\sqrt{\left[\frac{\sum {\left(0-x\right)}^{2}}{\text{number of datapoints}}\right]} \end{array}$$

(2) $$\begin{array}{c} \text{APSI}=\sqrt{\left[\frac{\sum {\left(0-y\right)}^{2}}{\text{number of datapoints}}\right]} \end{array}$$

(3) $$\begin{array}{c} \text{VSI}=\sqrt{\left[\frac{\sum {\left(\text{bodyweight}-z\right)}^{2}}{\text{number of datapoints}}\right]} \end{array}$$

(4) $$\begin{array}{c} \text{DPSI}=\sqrt{\left[\frac{\sum {\left(0-x\right)}^{2}+\sum {\left(0-y\right)}^{2}+\sum {\left(\text{bodyweight}-z\right)}^{2}}{\text{number of datapoints}}\right]} \end{array}$$

#### 2.3.3. Statistical Analysis

All outcome variables calculated in this study were presented as mean and standard deviation using the SPSS 26.0 (IBM, Chicago, IL USA) software for Windows. Normality assumption was first checked with the Shapiro–Wilk test (*p* > 0.05). The differences in kinematic and kinetics variables between the groups were analyzed using independent sample *t*-tests, and the kinematic variables influencing DPS were identified using stepwise multiple linear regression. Goodness of fit of the model is presented as the adjusted multiple coefficients of determination (*R*^2^). Coefficients (*R*^2^) were interpreted as weak (0.00–0.40), moderate (0.41–0.69), or strong (0.70–1.00). An *α* level is for all analyses was set at .05. Statistical significance level was set at *p* < .05.

## 3. Results

### 3.1. Kinematics and Kinetics Variables

The kinematic results of lower extremity joint angles and the kinetics results were compared at the time of mGRF. Except for knee internal rotation and ankle eversion, the two groups differed significantly across all variables. When compared with the control group, the PFPS group had significantly less hip flexion, internal rotation, knee flexion, and ankle external rotation and significantly more hip abduction, knee valgus, and ankle plantarflexion. There was a significant difference in mGRF, and there was no significant difference in leg stiffness. Compared with the control group, the mGRF of the PFPS group was significantly smaller (Table 2).

### 3.2. DPSI Results

DPSI was compared between the groups. The PFPS group had significantly greater APSI but significantly lower MLSI compared to the control group (Table 3).

### 3.3. Linear Regression Analysis of DPSI

Stepwise linear regression analysis was used to examine the effects of the landing motion on DPSI changes. In the control group, has been explained as having a negative effect on APSI (*R*^2^_(abj)_ = .198, *y* = 0.007 − 7.422^−5^*x*, Figure 3(a)), while knee internal rotation has been explained as having a positive effect on MLSI (*R*^2^_(abj)_ = .186, *y* = 0.014 + 5.927^−5^*x*, Figure 3(b)). In the PFPS group, ankle plantar flexion was explained to have a positive effect on MLSI (*R*^2^_(abj)_ = .302, *y* = 0.009 + 0.0001*x*, Figure 4).

## 4. Discussion

This study compared kinematics and kinetics variables and DPS during single-leg landing between the PFPS and control groups and used regression analysis to examine the effects of landing movement on DPS. We aimed to understand the kinetic features of lower limb joints and joint coordination during single-leg landing, as well as the influence of each lower limb joint on the DPS during single-leg landing in adult women with PFPS, to present foundational data for developing education about correct landing posture in patients with PFPS. As a result, the joint angle of the lower extremities and mGRF showed a significant difference between the PFPS group and the control group. In terms of DPS, the anteroposterior and mediolateral angles of the PFPS group were significantly higher than the control group, and the variables affecting the DPS were also different.

During single-leg landing, the PFPS group had less hip flexion and internal rotation and a larger abduction angle than the control group. According to studies, women with PFPS overstrain their knee joints due to valgus and hip adduction and internal rotation during knee flexion, when flexing the knee joints, and have a weaker hip abduction due to hip abductor muscle weakness [28, 29]. Pollard et al. [30] reported that people who exhibit a small hip flexion during drop landing place a greater load on the frontal plane of the knee joint, which is consistent with our findings. Participants with a small hip flexion angle use a strategy involving the knee extensor muscle, rather than the hip extensor muscle, to alleviate the shock, implying that using the hip extensor muscle is necessary to effectively use hip flexion during landing [30]. Furthermore, patients with PFPS have a weakening of the hip abduction and external rotation force [31]. Activating the hip external rotator and extensor muscles may help prevent the exacerbation of PFPS.

According to Pollard et al. [30], women with a small knee flexion angle during landing have more knee valgus than the control group. These women are thought to have compensated for the shock inflicted during single-leg drop landing through the knee valgus, similar to the PFPS group in our study who showed small knee flexion patterns during landing. Furthermore, the PFPS group's knee valgus pattern during landing may impair the ability to maintain knee alignment due to increased internal patellofemoral pressure, which intensifies the load in a smaller contact area and potentially escalates the pressure on the patellofemoral joint [13, 32]. Additionally, individuals also have an abnormal joint position sense [33], emphasizing the importance of joint repositioning training.

To absorb the GRF produced during landing, the ankle joints must shift from plantarflexion to dorsiflexion, and such an elevation of dorsiflexion may promote the stability of landing [34, 35]. In this study, the PFPS group was found to use an unstable and limited landing strategy, with significantly greater plantarflexion and internal rotation angle during single-leg landing than the control group. This is consistent with previous findings that a small dorsiflexion angle is related to knee flexion during landing [36, 37]. Furthermore, the PFPS group in previous study appears to have had impaired shock absorption control, which is consistent with previous studies that attributed the significant reduction in sagittal plane angle during landing in women with PFPS compared to their healthy counterparts to an impairment in shock absorption control [38]. In this study, the mGRF of the PFPS group was smaller than control group, and there was no difference in leg stiffness. It is thought that the PFPS group adopted a landing strategy differently from the control group, such as knee valgus. Rather than that, shock absorption was not properly controlled.

In terms of DPSI, the PFPS group had a higher APSI than the control group. PFPS causes quadriceps femoris and hamstring weakness, which results in an anterior displacement of the COP at peak GRF during landing [19, 39]. Patients with PFPS have severe anteroposterior instability, and inducing knee extensor fatigue increases anteroposterior instability [40]. Furthermore, the PFPS group had a low MLSI, which may be related to decreased control over knee movement due to knee valgus and pain [13]. A previous study found that the PFPS group had less COP displacement during a single-leg squat, and that a 9-week physical therapy intervention reduced pain while increasing COP displacement [41]. However, because it is unclear whether DPS is associated with knee movement and the motion characteristics may differ depending on the experimental task, further research on DPS is required [42, 43].

In this study, we used stepwise multiple regression to determine which kinematic variables best predict DPS. Knee flexion predicted APSI negatively while knee internal rotation predicted MLSI positively in the control group. A small amount of maximal knee flexion during landing may increase the shock to the lower limbs, and studies have shown that this is a poor landing strategy [44, 45]. Previous studies have found that stronger knee flexor and extensor muscles, as well as better proprioception, result in a greater knee flexion angle at initial grounding [46]. In another study, four weeks of plyometric and core training resulted in increased knee flexion and decreased internal rotation, which were attributed to lower knee joint loads [47]. Our findings suggest that increasing knee flexion while decreasing internal rotation is a strategy that promotes stability.

In the PFPS group, ankle plantarflexion was a positive predictor of MLSI, with MLSI increasing as ankle plantarflexion increased. Fong et al. [48] found that a small passive ankle dorsiflexion range of motion (ROM) can lead to large plantarflexion at landing, statistically significant high GRF and knee valgus, and small knee flexion, in a study on the correlation between passive ankle dorsiflexion ROM and landing. Furthermore, single-leg landing with a fatigued leg increases ankle plantarflexion and knee flexion, which is a compensatory strategy for fatigue-induced balance impairment and muscle weakness [34]. The PFPS group had large ankle plantarflexion and small knee flexion at peak GRF in this study, which can be attributed to the use of an ankle strategy during landing due to impaired knee motor control.

## 5. Limitation

The limitations of this study are as follows. Practicing single-leg drop landings for 15 minutes prior to the experiment may have affected the individual's pain level in this experiment. The control group may not have been affected, but the PFPS group may have been affected by the pain and landed with strategy to minimize the impact on the knee. In this study, the patellofemoral joint compression force was not measured directly, but was implied by the knee joint flexion angle. Further investigation in this area is needed in future studies. As a way to improve the landing strategy of the PFPS group, it may be helpful to practice the landing motion itself, which not only improves muscles strength but also improves coordination of the lower extremities.

## 6. Conclusions

This study observed that the PFPS group sustained more shock on their knees during landing compared to the control group. Also, while the control group used the knee and hip joint in the landing strategy, the PFPS group used the ankle strategy to compensate for the small flexion angle of the knee and hip joint. Individuals with PFPS use an unstable landing strategy, which causes an imbalance among the lower limb joints and raises knee pressure. To avoid this, the hip abductor, external rotator, and extensor muscles must be strengthened to allow for hip flexion. Furthermore, strategies for strengthening ankle dorsiflexion and activating the knee and hip flexors are required to correct the ankle-based landing strategy, and joint repositioning training should be performed to prevent pressure build-up due to abnormal joint position. In summary, it will be helpful to selectively classify the occurrence of PFPS through the analysis of the landing motion of adult women in this study and to develop rehabilitation training focusing on PFPS.

## Figures and Tables

**Figure 1:** Reflective marker attachment. (a) Static posture marker. (b) The four medial markers for movement have been removed.

**Figure 2:** Point of maximum ground reaction force during single-leg drop landing.

**Figure 3:** Results of linear regression analysis to normal group. (a) Results of linear regression analysis to normal group APSI. (b) Results of linear regression analysis to normal group MLSI. Abbreviations: APSI: anteroposterior stability index; MLSI: mediolateral stability index; adj: adjusted.

**Figure 4:** Results of linear regression analysis to PFPS group; results of linear regression analysis to PFPS group MLSI. Abbreviations: PFPS: patellofemoral pain syndrome; MLSI: mediolateral stability index; abj: adjusted.

**Table 1:** Characteristic of participants.

Variables	PFPS group (*n* = 19)	Normal group (*n* = 19)	*p*
Age (years)	23.11 ± 2.56	23.32 ± 2.24	.789
Height (cm)	163.42 ± 4.65	164.00 ± 4.78	.707
Weight (kg)	58.68 ± 7.61	55.08 ± 7.06	.139

Note: data are mean ± standard deviation. Abbreviations: PFPS: patellofemoral pain syndrome.

**Table 2:** Results of kinematics and kinetics at maximum ground reaction force.

Variables			PFPS group	Control group	*t*	*p*
Kinematics (°)	Hip	Flexion	11.262 ± 10.058	32.314 ± 9.786	-6.539	≤.001^∗∗∗^
		Abduction	14.802 ± 5.319	5.219 ± 4.283	6.117	≤.001^∗∗∗^
		Internal rotation	−7.459 ± 17.379	6.909 ± 9.787	-3.140	.003^∗∗^
	Knee	Flexion	18.775 ± 8.986	28.846 ± 8.634	-3.523	.001^∗∗^
		Valgus	−2.674 ± 5.939	−7.986 ± 5.219	2.929	.006^∗∗^
		Internal rotation	−10.944 ± 13.740	−11.547 ± 13.067	.139	.891
	Ankle	Plantarflexion	19.771 ± 6.974	8.725 ± 5.021	5.602	≤.001^∗∗∗^
		Internal rotation	6.129 ± 7.214	−1.788 ± 7.389	-3.342	.002^∗∗^
		Eversion	−13.808 ± 8.495	−11.016 ± 10.067	-.924	.362
Kinetics		mGRF	2.742 ± 0.817	4.432 ± 0.470	-7.815	≤.001^∗∗∗^
		Leg stiffness	27.680 ± 8.968	33.118 ± 8.993	-1.866	.070

Note: data are mean ± standard deviation. ^∗∗^*p* < .01, ^∗∗∗^*p* < .001; abbreviations: PFPS: patellofemoral pain syndrome; mGRF: max ground reaction force; “+” is the movement on the table, and “–”is the opposite movement (+: flexion, abduction, internal rotation, valgus, plantarflexion, and eversion; -: extension, adduction, external rotation, varus, dorsiflexion, and inversion).

**Table 3:** Results of dynamic stability index.

Variables	PFPS group (*n* = 19)	Normal group (*n* = 19)	*t*	*p*
APSI	.007 ± .002	.005 ± .001	3.240	.003^∗∗^
MLSI	.012 ± .002	.013 ± .002	-2.956	.005^∗∗^
VSI	.017 ± .009	.019 ± .010	-.956	.345
DPSI	.035 ± .011	.037 ± .010	-.713	.480

Note: data are mean ± standard deviation. ^∗∗^*p* < .01; abbreviations: PFPS: patellofemoral pain syndrome; APSI: anteroposterior stability index; MLSI: mediolateral stability index; VSI: vertical stability index; DPSI: dynamic postural stability index.

## Data Availability

The experiment data used to support the findings of this study are available from the corresponding authors upon request.
